# Simulation of Logistics Delay in Bayesian Network Control Based on Genetic EM Algorithm

**DOI:** 10.1155/2022/6981450

**Published:** 2022-04-07

**Authors:** Pengliang Qiao

**Affiliations:** ^1^School of Management, Guangzhou College of Technology and Business, Foshan 528138, Guangdong, China; ^2^School of Economics and Management, Beibu Gulf University, Qinzhou 535011, Guangxi, China

## Abstract

With the continuous development of e-commerce, the logistics industry is thriving, and logistics delays have become an issue that deserves more and more attention. Genetic EM algorithm is a genetic EM algorithm that is an iterative optimization strategy algorithm that can be used to solve the high-quality algorithm of travel problems with many nodes. Bayesian network (BN) is a network model based on probabilistic uncertainty. This article aims to study the probability of many factors that cause logistics delays to construct an algorithm model to control or reduce logistics delays. This paper constructs an EY model (That is the abbreviation of BN model based on genetic EM algorithm) based on the genetic EM algorithm, and conducts related simulation experiments based on the model to verify the accuracy and feasibility of the model. The experimental results of this paper show that the calculation efficiency of the EY model is significantly improved, and the actuarial accuracy is as high as 98%, which can effectively control logistics delays.

## 1. Introduction

### 1.1. Background and Significance

The concept of “logistics” varies from country to country and time to time. Generally speaking, logistics means the circulation of goods. The earliest logistic activity was recorded in the UK. The purpose at that time was to deliver the products to wholesalers, retailers and users nationwide in a timely manner. During World War II, the United States took military needs as the starting point and first adopted the term “logistics management” to refer to the supply of weapons during the war. In today's e-commerce era, the global logistics industry is experiencing new developments. The central goal of modern logistics services is to meet customer needs with the lowest comprehensive cost in the entire logistics process. However, with the rapid development of e-commerce, online shopping users' complaints about logistics delays have increased year by year. After analyzing the reasons in detail, it is found that the current solution to logistics delays is an urgent and resource-intensive emergency solution. This plan is incompatible with the normalization and globalization of e-commerce logistics packages. Therefore, it is necessary to have a deep understanding of e-commerce logistics, and formulate accurate measures based on scientific law analysis.

With the popularization of e-commerce now, logistics not only brings a lot of inconvenience to transportation, but once it is delayed, it will be subject to complaints from many customers and even large claims from partners. Studying how to control logistics delays and effectively avoid losses caused by logistics can not only reduce the complaint rate and improve customer satisfaction but also gain the trust of partners and win more cooperation opportunities, which is of great commercial significance.

### 1.2. Related Work

With the continuous development of the Internet of Things technology and the continuous prosperity of the logistics industry, more and more adults have conducted relevant research and exploration on logistics delays. With the development of the logistics industry, road traffic has become more and more congested. Due to the continuous changes in road conditions, the unstructured traffic chaos, the lack of lane discipline, and the wide variety of vehicles, there is a special need to develop a new type of traffic monitoring system. Chaudhary S uses dynamic BN to learn the pattern of road conditions and predict future road traffic conditions within a specific time delay. The predicted road condition information can be used for traffic planning. The method proposed by Chaudhary et al. is computationally lightweight, but very powerful and efficient. The algorithm has also been tested against various weather conditions. Chaudhary et al. uses Synchro Studio simulator (a traffic simulation software) to verify the algorithm, the average accuracy rate is 95.7%, for real-time video, the experimental accuracy rate is 84% [1]. Subjective detection is a natural language processing task designed to remove “facts” or “neutral” content from online product reviews, or objective text that does not contain opinions. Chaturvedi extends the extreme learning machine (ELM is a type of machine learning system or method based on feedforward neural network, suitable for supervised learning and unsupervised learning problems) paradigm to a new framework that uses the features of Bayesian and fuzzy recurrent neural networks to perform subjective detection. In particular, BN is used in the traditional ELM configuration to establish a network of connections between hidden neurons. The experimental results of Chaturvedi et al. verified the ability of the proposed framework to deal with standard subjective detection problems, and proved its ability to solve the portability between languages in translation tasks [2]. The multidimensional BN classifier is a topology-constrained BN, specifically used to classify data instances into multidimensional. Bolt and van der Gaag introduces the concept of balanced sensitivity function, in which multiple parameters are related in function by the odds ratio of the original value and the new value. These functions provide appropriate inspiration for adjusting the multidimensional classifier (It is a classification model that describes the dependency between class variables and class variables, class variables and attribute variables, and attribute variables and attribute variables) and output probability. The practical application of Bolt's classifier in the veterinary field proves the practicality of the heuristic method [3]. In ship reliability engineering, reliability evaluation is an important step to determine whether a ship has an acceptable level of reliability. Current reliability assessment methods are based on static logic. However, warships are typical power systems, and reliability cannot be evaluated by the above methods. Liang et al. proposed a new reliability evaluation method based on dynamic BN and numerical simulation. It overcomes the limitations of analysis methods and multi-level integration methods, and provides an effective means for evaluating ship reliability [4]. Based on dynamic BN with incomplete time slices and mixed Gaussian output, Zhang et al. proposed a data-driven method for predicting process failures with unknown models. According to the requirements of failure prediction, this method constructs an incomplete time slice BN of unknown future observation node. The method proposed by Zhang et al. is suitable for continuous stirred tank reactor system. The results show that even if some measured values are lost, the method proposed by Zhang et al. can effectively predict and identify faults and estimate the remaining service life of the process [5]. The original BN model did not have the expected variable hierarchy. When modeling the relationship between product sales in the retail industry, it is best to consider the hierarchy of items. Kawabe et al. proposed a hierarchical BN model based on the maximum and minimum hill climbing learning algorithm and a new learning method. The method proposed by Kawabe et al. focuses on the product hierarchy and allows the construction of a lower layer that considers the causality of the upper layer. In addition, Kawabe et al. investigated case studies using actual hierarchical data of consumer purchases and demonstrated the proposed model using simulation analysis [6]. Legal scholars have put forward examples of reasoning problems such as the twin problem and the poison paradox (that is, both the idea of drinking medicine and the cancellation of the idea of drinking medicine must be generated, which violates the law of contradiction) to prove the limitations of probability theory in legal reasoning. Specifically, such questions are intended to show that the use of probability theory may lead to legal paradoxes. Therefore, these problems have seriously affected the application of probability theory in law, especially Bayes' theorem. If various related hypotheses and evidence are correctly described in BN, the paradox disappears. Jacob demonstrated this with examples of food trays, the abuse paradox, and the murder problem in small towns. The resulting BN provides a powerful framework for legal reasoning [7]. However, the above research either lacks actual testing, or the calculation process is too complicated or even accurate, and it is currently difficult to pass.

### 1.3. Innovation

(1) The use of genetic EM algorithm can perform convergence calculations (it refers to the solution that has been numerically calculated, and if it continues to iterate, the result will not change) on unknown parameters, which can reduce logistics delay time. (2) Using BN to represent the graphical model of the connection probability of a set of variables, it provides a method for calculating logistics delays. (3) The EY model combined with the genetic EM algorithm and BN can greatly reduce the calculation error. (4) Comparing the EY model in this article with the traditional calculation model can better reflect the advantages of this model.

## 2. BN Model Based on Genetic EM Algorithm

### 2.1. Genetic EM Algorithm

1. The concept of genetic EM algorithm. The full name of genetic EM algorithm is Electromagnetic-like Algorithm, which is similar to electromagnetic mechanism algorithm. This algorithm is a new global improvement algorithm based on the meta-heuristic of group randomness. The earliest inspiration for this algorithm comes from the movement of point charges and Coulomb force in physics, as shown in. The genetic EM algorithm formulates criteria such as total force calculation between strokes, stroke power calculation, stroke motion, local search, etc., so that each stroke in the population moves in the direction of the optimal stroke, which can be obtained after repeated several times. The optimal solution of the optimization problem can be used as an independent algorithm to solve the global optimization problem. It can also be integrated with other algorithms to form a new global optimization algorithm (global optimization algorithm, also known as modern heuristic algorithm, is an algorithm with global optimization performance, strong versatility and suitable for parallel processing) [8].
2. Genetic EM algorithm classification. Because the genetic EM algorithm is a relatively new algorithm, domestic scholars have done very little research on the genetic EM algorithm, and the application of this method to the field of logistics distribution route optimization is still a blank. Fortunately, many researchers have done a lot of research on other optimization algorithms, including more advanced algorithms such as ant colony algorithm (it is a probabilistic algorithm used to find an optimal path, which comes from the behavior of ants finding paths in the process of looking for food) and genetic algorithm. Some scholars also apply these algorithms to the optimization problem selection of vehicle distribution routes, and have achieved certain results [9, 10].
3. The principle of genetic EM algorithm. Genetic EM algorithm is an iterative optimization strategy. The genetic EM algorithm is affected by the idea of data loss. It was originally to solve the problem of parameter estimation in the case of missing data. The basis and convergence of the algorithm are effective. The basic idea is as follows: first, estimate the value of the model parameters based on the given observation data. Then estimate the value of the missing data based on the parameter value estimated in the previous step, and then add the missing data previously estimated based on the estimated missing data. Re-estimate the parameter values from the observed data, and iterate repeatedly until the final convergence, and the iteration ends. Taking the question in this article as an example, assuming that the logistics has to pass through *k* nodes, then there are (*k* − 1)! ways to move, so how to make the logistics journey the shortest?

First, Figure 1 randomly selects a point from the known feasible region as the initial stroke, calculate the objective function *G*(*x*) of each stroke in a initial stroke, and calculate the optimal stroke *S*^𢄗^ of the objective function as the current optimal journey. Then set the local search parameters. Local search refers to an improved solution for searching the current population within a single travel range. According to the set local search parameters, calculate the various dimensions of the stroke, obtain the movement direction of the stroke and the maximum feasible step length, and perform a local search along this direction until a better solution is found. After the local search is completed, the population is updated once, the objective function value of each trip after the population update is recalculated, and the optimal trip of the objective function is updated. Then calculate the charge of each stroke according to the value of the objective function of each stroke, and then calculate the resultant force of each stroke through the formula of simulating electromagnetic field force and the principle of superposition. In the process of calculating the resultant force, the value of the objective function of each stroke is greater than the value of the objective function of the other two strokes. In this case, the (good) stroke with a small objective function value absorbs the stroke with a large objective function value, and the stroke with a large objective function value (bad) rejects the stroke with a small objective function value. The final stroke moves in the direction of the resultant force, and the feasible step length of each step of the stroke can be calculated by the following formula. At this time, the position of each stroke is updated, and the iteration of similar electromagnetic algorithms is completed [11, 12].

### 2.2. Bayesian Network

(1) *Concept.* Bayesian network (BN), also known as causal probability network and belief network, is a network model for reasoning based on probabilistic uncertainty, as shown in. The basis of BN is Bayes' theorem (A theorem about the conditional probability of random events *A* and *B*, where *P*(*A*|*B*) is the probability that *A* will occur if *B* occurs). BN is a network composed of nodes representing variables (including child nodes and parent nodes) and directed edges connecting these nodes. Random variables are represented by nodes, and the directed edges between each node represent nodes. The strength of the relationship is determined by the conditional probability. If there is no parent node, the information is represented by a priori probability. BN is a directed graphic description based on the network structure. This is a graphic model used to express the connection probability of a set of variables. It is suitable for expressing and analyzing uncertain and probabilistic things. It cannot be incomplete or uncertain, and must be based on knowledge and information. BN is a directed acyclic graph (A directed acyclic graph refers to a directed graph without a loop. If there is a non-directed acyclic graph, and starting from point A to B via C, it can return to A, forming a ring. Changing the edge direction from C to A from A to C becomes a directed acyclic graph. The number of spanning trees of a directed acyclic graph is equal to the in-degree product of nodes with non-zero in-degree.), and the acyclic graph (DAG) is composed of variable nodes and directed edges connecting these nodes [13, 14].
BN is a mathematical model based on random reasoning, as shown in Figure 2. The emergence of BN is to solve the problem of imperfection and uncertainty. This method helps to solve the uncertainty and correlation of complex equipment, and has great benefits for reducing risks. Probability theory is the theoretical basis of BN and an accurate solution to problems in probability theory. The BN theoretical system often uses some basic probability formulas, such as conditional probability, probability law, total probability, Bayesian formula, etc. [15].
(2) *Features*. BN can qualitatively express complex causal or random relationships between events in a concise graphical way. With some prior information, these relationships can also be expressed quantitatively. The topology of the network is usually determined based on specific survey topics and questions. One of the current research hotspots of BN is how to automatically determine and optimize the network topology through learning [16].
(3) *Bayesian Formula*. In order to solve the joint probability problem, there are usually different calculation methods for different probability events. The following are several common probability calculation formulas, in which the probability value is represented by *p*.
  (i) *Multiplication Formula*. If *X* and *Y* are two of the basic probability events of event *Z*, and the probability of any of these events is not 0, the calculation formula:
    (1) $$\begin{array}{c} p\left(XY\right)=p\left(X\right)p\left(Y|X\right), \end{array}$$
    (2) $$\begin{array}{c} p\left(XY\right)=p\left(Y\right)p\left(X|Y\right). \end{array}$$
  (ii) *Conditional Probability*. If *X* and *Y* are two of the basic probability events of event *Z*, there is a conditional relationship between the occurrence of event *X* and event *Y*, and the probabilities affect each other. If event *X* occurs and the probability is not 0, then the probability of event *Y* occurs:
    (3) $$\begin{array}{c} p\left(Y|X\right)=\frac{p\left(XY\right)}{p\left(X\right)}. \end{array}$$
  Similarly, if event Y occurs and the probability is not 0, then the probability of event *X*: Figure 2.
    (4) $$\begin{array}{c} p\left(X|Y\right)=\frac{p\left(XY\right)}{p\left(Y\right)}. \end{array}$$
  (iii) Using the multiplication formula and the conditional probability formula to generalize the total probability formula of the big event *Z*, assuming that *K*_1_, *K*_2_,…, *K*_*n*_ are the sub-events of event *Z*, and the probability of occurrence of the event is not 0, then the total probability formula of event *Z* can be expressed as:
    (5) $$\begin{array}{c} p\left(Z\right)=\overset{n}{\underset{i=1}{\sum }}p\left(K_{i}\right)p\left(Z|K_{i}\right). \end{array}$$
  From this, the conditional probability formula of the event *K*_*i*_ can be scored:
    (6) $$\begin{array}{c} p\left(Z|K_{i}\right)=\frac{p\left(Z\right)}{\sum_{i=1}^{n}p\left(K_{i}\right)}. \end{array}$$
  (iv) *Bayesian Formula*. Assuming that *K*_1_, *K*_2_,…, *K*_*n*_ are the sub-event groups of event *Z*, the probability is not 0, and the event *X* is any event among them, and the probability is not 0, then the above generalization can be obtained:
    (7) $$\begin{array}{c} p\left(K_{i}|X\right)=\frac{p\left(K_{i}\right)p\left(X|K_{i}\right)}{\sum_{j=1}^{n}p\left(K_{j}\right)p\left(X|K_{j}\right)}. \end{array}$$
(4) *BN Mathematical Model*. BN modeling is a relatively complicated process, which requires patience and care. When modeling, the first thing to do is to determine the nodes, use the nodes to build the topology, then calculate the conditional probability distribution of each node, and finally test to determine the model. shows the basic model building process [17, 18].
  (i) Selection of nodes. Bayesian network node variables are various elements of the emergency system. It is very important to determine the node variables as comprehensively as possible for the accuracy of situation assessment. There are several main types of nodes in Bayesian networks. The first is the target node. This node represents the final problem that the model needs to solve. The second is the evidence node (also called the parent node), which is the most basic parent node in the network and has a value similar to the following: the prerequisites for Bayesian network inference are provided directly from the database or provided by expert knowledge. The third is to realize a component of the integrity of the Bayesian network. After determining the connected role nodes, the value of each node needs to be further determined. The value of each node is independent of each other and does not contain each other [19].
  Assuming that there are *m* nodes in BN, and each node is represented by *N*, then: Figure 3.
    (8) $$\begin{array}{c} P\left(N\right)=P\left(N_{1},...,N_{m}\right). \end{array}$$
  Taking *m* equal to 4 as an example, suppose there are four nodes *H*, *I*, *J*, and *K*, as shown in Figure 4:
  According to the previous probability formula, we can get:
    (9) $$\begin{array}{c} P\left(H,I,J,K\right)=P\left(K|J\right)|P\left(I|H,J\right)|P\left(J|H\right)|P\left(H\right). \end{array}$$
  (ii) The establishment of BN topology. The purpose of BN structure learning is to extract specific data and build a structure with a higher degree of fit. According to the previous knowledge, when the number of nodes is *m*, the number of structures can be expressed as a function:
    (10) $$\begin{array}{c} G\left(m\right)=\overset{m}{\underset{i=1}{\sum }}{\left(-1\right)}^{i+1}\left[\frac{m!}{i!\left(m-1\right)!}\right]2^{i\left(m-1\right)}g\left(m-i\right). \end{array}$$
  Using the scoring search method to perform statistics, *R* represents random variables, and *S* represents data collection, then:
    (11) $$\begin{array}{c} R=\arg\max P\left(R|S\right), \end{array}$$
    (12) $$\begin{array}{c} P\left(R|S\right)=\frac{P\left(S|R\right)|P\left(R\right)}{P\left(S\right)}. \end{array}$$

According to formula (12), the logarithm of both sides can be obtained

(13) $$\begin{array}{c} \text{Log}P\left(R|S\right)|=\text{Log}P\left(S|R\right)|+\text{Log}P\left(R\right). \end{array}$$

Formula (13) is the score of *R*. In fact, *P*(*R*) is usually evenly distributed, for which one can obtain

(14) $$\begin{array}{c} P\left(S|R\right)=\int P\left(S|R,\delta \right)|P\left(\delta |R\right)|d\delta . \end{array}$$

In the formula, *δ* represents the size of the node corresponding to *R*.

When the data set *S* is independent and identically distributed, and *R* is the corresponding BN structure, the evaluation function for BD is

(15) $$\begin{array}{c} G_{BD}\left(R,S\right)=\text{Log}P\left(R\right)+\overset{m}{\underset{i=1}{\sum }}\overset{h_{i}}{\underset{j=1}{\sum }}\left[\text{Log}\frac{\Gamma \left(x_{i,j}\right)}{\Gamma \left(x_{ij*}+y_{ij*}\right)}+\overset{d_{i}}{\underset{c=1}{\sum }}\frac{\Gamma \left(x_{ijc}+y_{ijc}\right)}{\Gamma \left(x_{ijc}\right)}\right]. \end{array}$$

When the data set *S* is independent and identically distributed, and *R* is a BN structure of *y* variables, the evaluation function for K2D is

(16) $$\begin{array}{c} G_{K2}\left(R,S\right)=\text{Log}P\left(R\right)+\overset{m}{\underset{i=1}{\sum }}\overset{h_{i}}{\underset{j=1}{\sum }}\left[\text{Log}\frac{\left(d_{i}-1\right)!}{\left(y_{ij}+d_{i}-1\right)!}+\overset{d_{i}}{\underset{c=1}{\sum }}\text{Log}\left(y_{ijc}\right)\right]. \end{array}$$

If the BN structure information is uniformly distributed, the evaluation function for BDe is

(17) $$\begin{array}{c} G_{B\;De}\left(R,S\right)=\text{Log}P\left(R\right)+\overset{m}{\underset{i=1}{\sum }}\overset{h_{i}}{\underset{j=1}{\sum }}\left[Log\frac{\Gamma \left(x/h_{i}\right)}{\left(\Gamma \left(x/h_{i}\right)+y_{ij*}\right)}+\overset{d_{i}}{\underset{c=1}{\sum }}\frac{\Gamma \left(\left(x/d_{i}h_{i}\right)+y_{ijc}\right)}{\Gamma \left(x/d_{i}h_{i}\right)}\right]. \end{array}$$

Or an evaluation function based on information theory, *LL*(*R*|*S*) represents the logarithm of the likelihood of BN, then

(18) $$\begin{array}{c} G\left(R|S\right)=g\left(\delta \right)\left|R\right|-LL\left(R|S\right). \end{array}$$

When *g*(*δ*)=1, there are

(19) $$\begin{array}{c} G_{A}\left(R|S\right)=\left|R\right|-LL\left(R|S\right). \end{array}$$

When *g*(*δ*)=(1/2)Log*m* represents the number of bytes

(20) $$\begin{array}{c} G_{B}\left(R|S\right)=\frac{1}{2}\text{Log}\left|R\right|-LL\left(R|S\right). \end{array}$$

The selection of the evaluation function should be carried out according to the actual situation of the BN network, and the minimum evaluation function obtained by calculation can obtain the best parameters of BN [20, 21].

### 2.3. Plan to Control Logistics Delays

#### 2.3.1. The Meaning of Logistics Delay

The rapid development of e-commerce has brought more and more convenient online shopping services, and at the same time, it has also driven the rapid development of the logistics industry. shows the growth of online shopping users and the amount of online shopping transactions in the past five years.

It can be seen from Figure 5 that with the continuous development of e-commerce, the number of online shopping users has increased year by year, and the total amount of e-commerce transactions has also continued to increase. Due to the impact of the epidemic at the end of 2019, its online shopping transaction volume has declined, but online shopping users are still increasing, which also shows that during the epidemic, more and more people began to prefer online shopping. Figure 5.

However, there are also a lot of problems in the development process of the logistics industry. As a service-oriented industry, logistics is the most important thing to ensure the timely delivery of goods, so the problem of logistics delays is the most worthy of attention.  Figure 6 shows the growth of the express delivery industry in recent years and the growth of the number of complaints about logistics delays by express users to the State Post Bureau.

It can be seen from Figure 6 that the number of complaints about logistics delays by express users to the State Post Bureau has been increasing year by year, and the number of express delivery delays accounted for more than 25% of the total number of complaints, such a serious delay has brought a lot of discomfort to e-commerce merchants, operators and users. For e-commerce merchants, delays in e-commerce logistics have brought them credibility and economic losses. Major e-commerce platforms regard logistics as an indicator for customers to evaluate their online stores. The poor experience of logistics delays will affect the reputation of the customer's store, damage the reputation of the store, and affect the decision of other potential customers whether to purchase the store's goods [22, 23].

#### 2.3.2. Reasons for Logistics Delays

According to the direct personnel contacting the goods, it can be divided into corporate factors (including logistics company factors, provider factors, courier factors), customer factors and other factors. Logistics company factors include arranging logistics drivers for loading, transportation schedules and other factors; providers include delivery speed, packing speed, etc.; the courier includes the speed of handover, telephone notification to customers, etc.; customer factors include pickup speed, fuzzy receiving address, incorrect phone number, etc.; other factors include road traffic conditions, weather factors, emergencies, and so on.  Table 1 shows the statistics of the proportions of various factors, among which the corporate factor is the most important factor.

#### 2.3.3. Features

When e-commerce logistics is delayed at the starting node, the delay will spread downstream through online shopping products. Affected by this, e-commerce logistics continues to lag downstream neighboring nodes, and there is a continuous delay between this point and downstream neighboring nodes. Affected by interference factors, there is a complicated correlation between the initial delay in e-commerce logistics at the starting node and the adjacent delay in downstream adjacent nodes. Initial delays in commercial logistics can increase, pass on, or weaken the impact of adjacent delays. Delivery companies have different factors in e-commerce logistics delay management methods, leading to the introduction of corporate and customer factors. The degree of correlation between successive delays in e-commerce logistics caused by various factors varies.  Figure 7 is a schematic diagram of the spread of logistics delays [24].

#### 2.3.4. Control Measures for Logistics Delays

Based on the analysis of the causes of logistics delays, it can be carried out from the aspects of enterprises, customers, etc., and other factors can be avoided if they can be avoided. On the corporate side, improvements or optimizations can be made in terms of employees, equipment, management methods, etc., while on the customer side, communication with them can be strengthened, and logistics awareness can be promoted. In other aspects, such as sudden traffic jams, if the transportation cost is similar, the detour is faster if it can take a detour. In severe weather, it can choose a better logistics method. ① In terms of corporate employees, improving the working level of the staff not only guarantees the work quality of the courier, but also ensures that the behavior of the customer during the delivery process meets the requirements of the courier, and avoids the delay caused by the following reasons in e-commerce logistics: operation error. Human factors are now an important reason for e-commerce logistics delays. Improving the work level of personnel is the key to avoiding unreasonable delays and an important means to control the spread of delays. To improve staff credibility, it is necessary to strengthen the training and management of express company employees. The staff of courier companies need to have professional knowledge and skills to effectively avoid delays caused by seal errors, misdelivery, and failures in timely response. At the same time, having professional knowledge and a sense of responsibility is an important guarantee for the courier staff to correctly guide the delivery behavior of customers and avoid problems such as blurred addresses and telephone errors. ② Stability of working equipment. The failure of logistics operation equipment is an important factor causing delays in e-commerce logistics. By improving the reliability of logistics equipment, it can effectively reduce the possibility of logistics delays caused by corporate factors in e-commerce. For this reason, this section focuses on the maintenance and repair management of logistics equipment. Working and deploying the correct logistics equipment are two aspects of improving equipment reliability. One is the regular maintenance and overhaul management of logistics equipment. The logistics company's regular maintenance and overhaul management of logistics equipment can effectively avoid delays caused by mechanical equipment failures, increase equipment reliability, reduce potential delays in the cradle, and provide guarantee for e-commerce logistics operation planning. The second is to introduce appropriate logistics equipment. The introduction of suitable logistics equipment by logistics companies can effectively improve the efficiency of logistics operations, reduce the actual operation time of e-commerce logistics, and increase the “slack time” in the logistics operation process. If there is a delay in e-commerce logistics, e-commerce logistics is one of the nodes. The longer the “relaxation time” between the two, the more helpful it is to absorb the delay time and reduce the spread of the delay. ③ Reasonably arrange the priority of logistics business. Due to corporate factors, enterprises have poor management of e-commerce logistics delays. The spillover effect of delays is mainly manifested in transmission, and the delay absorption rate is very low, which reduces customer satisfaction with carriers and shipments, and damages the company's reputation. If e-commerce logistics is delayed due to corporate factors, the company is fully responsible, and the company must have greater control over the increasingly serious logistics delay. This article recommends that companies adopt new business priority allocation to solve the problem of e-commerce logistics delays caused by corporate factors. That is, change the logistics route and choose the route with higher priority [25].

## 3. EY Model Logistics Delay Control Simulation Experiment

### 3.1. Design of EY Model

#### 3.1.1. Design Ideas

According to the number *m* of nodes passed by the logistics, the delay of each node logistics will affect the logistics delay of the two goods before and after, as shown in Figure 8, the entire logistics business process of online shopping from receipt to delivery is connected. The goods pass through *x*_1_, *x*_2_,…, *x*_*i*_,…, *x*_*m*_ logistics nodes in sequence according to the logistics plan. *i* is a positive integer. The delay of online shopping at specific logistics nodes will inevitably affect the timeliness of subsequent logistics nodes. In the process of logistics business, there is “logistics slack” in online shopping products. For example, an online shopping product will stay at a specific logistics node for an hour, but in reality, the staff of the logistics node will complete half of the logistics transfer activities such as weighing, loading and unloading, and product handling. The remaining 30 minutes are “logistics slack,” but “logistics slack” may not be enough to absorb the delay time of the product operation on the previous node, leading to the spread of delays. If the user suggests to the carrier that the delivery of online shopping goods from node *x*_*i*_ to node *x*_*i*_ + 1 is delayed, the goods will continue to pass through nodes *x*_*i*_, *x*_*i*_ + 1…*x*_*m*_ to the preliminary planned route of subsequent logistics business activities. Assuming that in the process of sending online shopping products from node *x*_*i*_ to node *x*_*i*_ + 1, the delay cannot be fully absorbed due to the interference factor “logistics slack,” then the arrival of online shopping products at node *x*_*i*_ + 1 will be delayed; if *x*_*i*_ + 1 is affected by the delay time of the node after receiving, “logistics slack” cannot fully absorb the remaining delay time in the processing of online shopping products from node *x*_*i*_ + 1 to node *x*_*i*_ + 2, online shopping arrival delay node *x*_*i*_ + 2 products will certainly continue to be delayed. This paper mainly studies the delay propagation of online shopping products from node *x*_*i*_ + 1 to delivery node *x*_*n*_. Node *x*_*i*_ + 1 is defined as the starting node and node *x*_*i*_ + 2 is the adjacent node; the delay of online shopping products at the starting node is defined as the initial delay. The delay of online shopping products on adjacent nodes affected by the initial delay is defined as the adjacent delay. The delay of online shopping products affected by the initial delay is defined as the delay of the delivery node. The delay time of the online shopping product at the starting node is defined as the initial delay time, that is, the difference between the time when the online shopping product actually arrives at the starting node and the planned time. The node delay time when the online shopping product is adjacent is defined as the adjacent delay time, that is, the difference between the actual time and the planned time for the online shopping product to reach the adjacent node; the delay time of the online shopping product at the delivery node is defined as the total delay time. This is expressed as the difference between the actual time and the planned time for the online shopping product to arrive at the delivery node. Online shopping products are affected by initial delays in the distribution process, and online shopping products continue to reach downstream nodes. Delay nodes (except the start node) are defined as downstream delay nodes [26, 27].

Figures 7 and 8 original delay model is improved and simplified, and the EY model is obtained. The model comparison is shown in Figure 9. The numbers in the figure represent various causes of logistics delays. Figure (a) is the model before improvement, and figure (b) is the model after improvement.

#### 3.1.2. The Characteristics of the Improved Model

The streamlined model is smaller in scale, faster in calculation, and suitable for processing large data sets. The improved model combines related factors, its structure is clearer, the calculation path is clearer, there is no redundant calculation, the simplified model is smaller in scale, faster in calculation, and suitable for processing large data sets. In the logistics delay forecast, the effect is better and the accuracy rate is high.

### 3.2. Simulation Experiment of Logistics Delay Control Based on EY Model

This article simulates the simulation experiment of logistics transportation route optimization, and the selected EY model is feasible and efficient. Collecting data before the experiment. Before the experiment, this article investigated the complaints, data management, delayed mediation, problem handling, etc. from many domestic express company users. The data includes the number of courier services and delay factors for online shopping products. The selected courier tracking number is one of the courier's working group, indicating that the delayed item was purchased online, or the logistics information of the delayed item indicates that the seller shipped it. This article collected 11,000 e-commerce logistics delay data, of which 8,500 valid data. The number of e-commerce logistics delays caused by corporate factors was 6,213; the number of delays caused by customer factors was 2,101; and the number of e-commerce logistics delays caused by other factors was 186. As shown in Table 2.

The experiment selected 18 logistics nodes where a logistics company is about to transport goods. The purpose is to calculate a more reasonable logistics distribution route to make the transportation mileage the shortest. The logistics node is represented by two-dimensional coordinates (*i*, *j*), as shown in Table 3.

According to the permutation and combination algorithm, there are a total of 18 paths, including more than 6,400 trillion ways. It is basically difficult to calculate. Using the model optimization algorithm designed in this paper, first select a node as the center node, the coordinate center point is (100, 100), because considering that the node closest to the coordinate center point is the node number 15, the center node coordinate is selected as the number 15 (126, 85). According to the previous formula, take *m* as 18. After iterative calculation, the better mileage shown in Table 4 is obtained, and the corresponding comparison is shown in Figure 10.

The experimental results found that the calculation of the optimal route for the total mileage of the logistics transportation route calculated by the EY model has high accuracy, few iterations of the calculation, and high calculation efficiency. The optimal route obtained after 9 calculations is 1106 km. Among them, the number of occurrences of the optimal route is 4 times, ranking first. The longest calculation is 1225 km, the distance error is less than 1.1%, and the calculation accuracy is as high as 98%.

## 4. Discussion

The electromagnetic-like mechanism of logistics transportation path optimization algorithm simulates the mechanism of charged particles in physics, so that the particles move to the optimal solution. Particle turbulence allows the local search mechanism to search better both locally and globally. In order to obtain the best solution, the goal of preventing the best solution from slipping through the network has been achieved.

## 5. Conclusions

The EM algorithm proposed in this paper has made a certain breakthrough in solving the problem of logistics transportation route optimization. However, there is still room for further research on this issue. This article only conducted simulations with careful consideration of distance and calculation of increased vehicle restrictions and vehicle capacity restrictions. Road congestion is frequent in logistics and transportation, and short-distance routes will waste a lot of time due to congestion, resulting in reduced transportation efficiency. Therefore, in future research, it is necessary to increase congestion parameters and time parameters, comprehensively consider the length of the trip and the time of the trip, and obtain an algorithm that matches the actual logistics road conditions.

## Figures and Tables

**Figure 1:** Schematic diagram of EM algorithm.

**Figure 2:** BN model.

**Figure 3:** BN model establishment process.

**Figure 4:** BN structure model of four nodes.

**Figure 5:** The development of online shopping and express delivery in China in recent years. (a) Growth of online shopping users. (b) Growth of online shopping transactions.

**Figure 6:** The number of express complaints about logistics delays in recent years. (a) Growth in express delivery business. (b) Delay in express delivery complaints.

**Figure 7:** Schematic diagram of the spread of logistics delays.

**Figure 8:** Schematic diagram of logistics delays.

**Figure 9:** Logistics delay model.

**Figure 10:** Results of route calculation by EY model. (a) Node distribution map and (b) Calculate a high-quality roadmap.

**Table 1:** Proportion of reasons for logistics delays.

Factor	Include	Proportion (%)
Company	Logistics company	56.2
	Enterprise store	27.9
Customer	Pickup speed	11.6
Other	Natural factors	4.3

**Table 2:** E-commerce logistics delay data.

Genre	Number	Proportion (%)
Valid data	8500	77.27
Business delays	6213	73.09
Customer delays	2101	24.72
Other delays	186	2.19
Logistics delay total	11000	

**Table 3:** Distribution of logistics nodes.

Node code	*i*	*j*
1	116	9
2	104	19
3	70	132
4	179	139
5	159	62
6	5	94
7	176	85
8	145	24
9	173	175
10	127	165
11	72	140
12	83	31
13	35	117
14	21	142
15	126	85
16	17	19
17	23	196
18	67	123

**Table 4:** Calculation results of EY model.

Total distance (km)	Number of calculations	Route
1225	2	A
1106	4	C
1139	3	B

## Data Availability

No data were used to support this study.
